# Deep-Learning-Based CT Imaging in the Quantitative Evaluation of Chronic Kidney Diseases

**DOI:** 10.1155/2021/3774423

**Published:** 2021-10-28

**Authors:** Xu Fu, Huaiqin Liu, Xiaowang Bi, Xiao Gong

**Affiliations:** ^1^Second Department of Nephrology, Zibo Central Hospital, Zibo 255000, Shandong, China; ^2^Department of Radiology, Zibo Central Hospital, Zibo 255000, Shandong, China

## Abstract

This study focused on the application of deep learning algorithms in the segmentation of CT images, so as to diagnose chronic kidney diseases accurately and quantitatively. First, the residual dual-attention module (RDA module) was used for automatic segmentation of renal cysts in CT images. 79 patients with renal cysts were selected as research subjects, of whom 27 cases were defined as the test group and 52 cases were defined as the training group. The segmentation results of the test group were evaluated factoring into the Dice similarity coefficient (DSC), precision, and recall. The experimental results showed that the loss function value of the RDA-UNET model rapidly decayed and converged, and the segmentation results of the model in the study were roughly the same as those of manual labeling, indicating that the model had high accuracy in image segmentation, and the contour of the kidney can be segmented accurately. Next, the RDA-UNET model achieved 96.25% DSC, 96.34% precision, and 96.88% recall for the left kidney and 94.22% DSC, 95.34% precision, and 94.61% recall for the right kidney, which were better than other algorithms. The results showed that the algorithm model in this study was superior to other algorithms in each evaluation index. It explained the advantages of this model compared with other algorithm models. In conclusion, the RDA-UNET model can effectively improve the accuracy of CT image segmentation, and it is worth of promotion in the quantitative assessment of chronic kidney diseases through CT imaging.

## 1. Introduction

At present, chronic kidney disease has affected approximately 10% of the world's population, killing millions of people every year, and hundreds of thousands of people undergo dialysis to maintain their lives [1]. Chronic kidney disease refers to changes in the structure and function of the kidney that have occurred for more than three months. Renal cysts are one of them, but renal cysts are benign structural changes. Renal cysts grow slowly and will not have an impact on patients in the short term. However, as the cysts increase, they will compress the gastrointestinal tract. As a result, the volumes of the stomach and intestine shrink, and the patient will feel full all the time. Some patients also have symptoms of fever, vomiting, and abdominal pain, so they will have a negative impact on the patient's psychology and physiology [2–4]. During treatment, it is difficult to accurately distinguish renal cysts from small cystic renal cell carcinoma, which affects the formulation of appropriate treatment plans for patients [5]. Hence, finding a safe and reliable way to detect renal cysts is important for the treatment of patients. In clinical practice, X-rays, CT, and B-ultrasound are commonly used to diagnose patients with the kidney disease. CT scans a part of the human body with X-ray beams to obtain a cross-section or stereo image of the part being examined. It can provide complete three-dimensional information of the part of the body being examined, clearly displaying the organs and structures, as well as the lesions. The biggest advantage is that it can be viewed in layers so that more organizational information can be displayed after calculation [6]. Therefore, the application of CT in kidney examination is a hotspot of current research.

Deep learning is the core of artificial intelligence technology, and it is a research hotspot in recent years. In 2006, Dong first proposed the concept of deep learning. In order to optimize the deep structure, they proposed a greedy layer-by-layer training algorithm on the basis of the deep belief network [7]. Deep learning algorithms have also been widely used in medical image segmentation. Song et al. used the kernel fuzzy C-means algorithm and the improved GrowCut algorithm to segment kidney images, and the automatically generated seed labels heightened the segmentation efficiency [8]. Xiang et al. used cortical models and nonuniform maps to depict the kidney structure in CT images [9]. Xiong et al. proposed a tumor segmentation method based on adaptive partitioned firework level sets, which effectively segmented kidney tumors in ultrasound images [10]. Gao incorporated the level set into image segmentation to process images with uneven gray values and achieved good segmentation results [11]. Hu introduced the target tracking mechanism into the traditional image segmentation and achieved good segmentation results [12].

In this study, the U-shaped fully convolutional neural network (CNN) segmentation model was optimized by incorporating a residual dual-attention module to the model to elevate the accuracy of locating the edge of the cyst, thus to accurately and quantitatively assess chronic kidney diseases.

## 2. Experimental Principles and Methods

### 2.1. UNET Segmentation Model Based on the RDA Module

The RDA module is incorporated into the UNET model, so the optimized one is called RDA-UNET, and the structure is shown in Figure 1.

#### 2.1.1. RDA Module

Heet al. deepened the network by stacking residual units to ensure the integrity and safety of the information and reduce the learning difficulty [13]. Woo et al. proposed a convolution algorithm that combines the channel with spatial information to extract information features, but the convolutional features are messy, so the attention mechanism can only focus on meaningful features extracted from a certain dimension [14]. In this study, a residual attention module is proposed based on the residual unit structure and attention mechanism, as shown in Figure 2.

For the input image, after going through the convolutional operation twice in the RDA module, it is processed by the channel and spatial attention mechanism, and then elements are added to it, followed by the residual connection with the original image, and finally, it is processed by the ReLU function. The original image is *Y* ∈ *Ww* × *w* × *c*, *y* is the size of the image, and *C* is the number of channels. The specific process of the dual-attention mechanism is as follows. According to the position of the pixel, the spatial attention mechanism identifies its contribution, and then the 1 × 1 convolution and sigmoid activation function are used to calculate the single-channel spatial attention mask *Q* ∈ *Ww* × *w* × 1 of each position pixel. Then, the original image *Y* is multiplied with the single-channel spatial attention mask *Q*. For the channel spatial attention mechanism, the contribution of each channel is firstly identified, and then 1 × 1 convolution and sigmoid activation function are used to calculate out-channel attention code *P* ∈ *W*1 × 1 × *c*, and finally, the original image is multiplied by the channel attention code. The steps of the dual-attention mechanism can be expressed as follows:

(1) $$\begin{array}{c} Y^{\prime }=Q\left(Y\right)⊗Y+P\left(Y\right)⊗Y, \end{array}$$

where *Y*′ represents the output image, ⊗ represents element-wise multiplication, and *Q*(*Y*) and *P*(*Y*) represent the size same as *Y* in the channel and space, respectively. The RDA module has two advantages. One is to repeatedly use the features, and the other is the adaptive learning feature table. Hence, the module can learn the features of the image more effectively.

#### 2.1.2. RDA-UNET Network Structure

According to the structural characteristics of UNET, the RDA module is introduced to design a new deep segmentation model, and its network structure is shown in Figure 1. It is mainly composed of four parts of encoder, bottleneck layer, decoder, and classifier. The encoder mainly includes the RDA module and the maximum pooling layer. The main function is to extract the semantic features of the original image. The pooling layer is mainly used for image downsampling, so as to increase the neuron sensor to obtain more detailed semantic feature information. The bottleneck layer is mainly composed of two convolutional layers, which are mainly used during the transition from the encoder to the decoder. Two deconvolutional layers and an RDA template form the decoder part, which is mainly used for image feature reconstruction, and the deconvolution layer is used for upsampling to improve the resolution of the image. The classifier is composed of a convolution layer and a softmax layer. This part can be used to estimate the background image before and after. In this part, the convolution layer can reduce the number of channels. Softmax is used to calculate the probability of the pixel belonging to a certain category. In the decoder and encoder, images of the same level can be jump-connected, thus providing rich pixel-level information for feature reconstruction. In addition, zero-filling convolution is used in each convolutional layer to obtain feature maps of the same size. In order to prevent the gradient from rising and disappearing, BN is used for all convolutional layers (the parameter settings used by the encoder and decoder are similar).

The probability map is the ratio of each pixel on the kidney and not on the kidney. The loss function is obtained by manually labeling the mask and the probability map. In this study, Dice loss is used to optimize training [15]. Dice coefficient is to evaluate the similarity, which can be expressed as follows.

(2) $$\begin{array}{c} \text{Loss}=1-\frac{2\sum_{y}^{N}h_{i}\left(y\right)k_{i}\left(y\right)}{\sum_{y}^{N}h_{i}^{2}\left(y\right)+\sum_{y}^{N}k_{i}^{2}\left(y\right)}, \end{array}$$

where *N* represents the number of pixels, *h*_*i*_(*y*) represents the estimated probability that the *y*th pixel belongs to category *i*, and *k*_*i*_(*y*) represents the probability that the true *y*th pixel belongs to category *i*.

### 2.2. Experimental Settings

Dataset: the clinical abdominal plain CT images of patients with renal cysts were collected, and the images with obvious renal cyst lesions were manually marked by experienced experts. The data format is set to DICOM format, the distance between pixels is 0.625 mm, the thickness of image slices is generally 1.0 mm, and the distance between slices is about 0.5 mm. The resolution of Tuqiang is set to 512 × 512. A total of 79 patients with renal cysts were selected, and 6000 slice images were obtained. 27 cases were defined as the test group, and 52 cases were defined as the training group.

Preprocessing: the image needs to be processed before the experiment. First, the window width and window position of the image are adjusted to 420 hu and 60 hu, and then the size of the image is reduced to increase the number of images for each training. The image size is adjusted to 256 × 256. In order to make the network training more adequate, it is necessary to double the training set data by horizontal flipping. Finally, the image is normalized.

Hardware configuration and development environment: processor: Intel (R) Core(TM) i7-4790 CPU @ 3.60 GHz; discrete graphics card: Ge Force GTX Titan X; memory (RAM): 32.0 GB; system type: Ubuntu 16.04; development language: Python; deep learning framework: PyTorch [16]; image reading software: ITK-SNAP [17].

Parameter settings: batch size is set to 16; the initial learning rate is set to 10^−3^, and it is automatically set to 10^−4^ when 30 epochs are completed; the momentum is set to 0.95, and the weight attenuation coefficient is constant 10^−4^_._ The Adam optimizer is used for training, the training stops automatically after 50 epochs, and the test selects the parameter with the smallest loss value.

### 2.3. Evaluation Index

According to Figure 3, the kidneys are located on both sides of the spine. In this study, the spine was regarded as the dividing line, and the method of artificially annotating images and the method of network prediction were used to segment the left and right kidneys. Since the left and right kidneys are not at the same height, the image will display other parts except the kidneys. The parts will be deleted during manual labeling and grid prediction. The segmentation accuracy was evaluated factoring into DSC, recall, and precision, defined as follows.

(3) $$\begin{array}{c} \text{DSC}=\frac{2\left|E\cap F\right|}{\left|E\right|+\left|F\right|}, \end{array}$$

(4) $$\begin{array}{c} \text{precision}=\frac{SQ}{SQ+HQ}, \end{array}$$

(5) $$\begin{array}{c} \text{recall}=\frac{SQ}{SQ+HM}. \end{array}$$

In equation (3), the model prediction result is *E*, *F* is the corresponding manual labeling result, and *E*∩*F* represents the foreground part in the segmentation image. In equations (4) and (5), *SQ* represents the part of the kidney that is correctly predicted, *HQ* represents that the background is predicted as the kidney, and *HM* represents that the kidney is predicted as the background.

### 2.4. User Interface

In order to facilitate operations, a simple user interface was designed using the Tkinter module based on the RDA-UNET model. This interface can accurately infer the edge contour, assisting users in segmentation.

### 2.5. Principles of 3D Reconstruction

CT imaging can reconstruct the three-dimensional image of the kidney. The three-dimensional image can accurately locate the area where the kidney is located to extract effective information. Doctors can preliminarily diagnose the type, the size, and the area of the renal cysts through the three-dimensional image. In addition, studies [18] have shown that the total kidney volume (TKV) is associated with the renal function to a certain extent. The TKV can be estimated by reconstructing the three-dimensional image of the kidney, and then the severity of the disease is evaluated. Therefore, the three-dimensional image of the kidney is reconstructed in the study.

## 3. Results

### 3.1. Comparison of Segmentation Effects

Figure 4 shows the relationship between the loss function of the network model in this study and the number of iterations in the training process. It was noted that the value of loss function can quickly decay and converge when the Adam optimizer was used.

Figure 5 shows the segmentation results of some images and their visualization during the training process. It was noted that the segmentation results of the algorithm proposed in this study were roughly similar to the results of manual labeling, and the spatial attention mechanism effectively and adaptively learned the spatial features. On the test set, the evaluation indicators of network models of different depths are shown in Table 1. The original models mainly included FCN-8S, FCN-16S, U-Net, and FCN-VGG10. On the basis of U-Net, U-Net (+BN) model was obtained, and UNet++ was further obtained on the basis of U-Net (+BN). In order to ensure the fairness of the experiment, no in-depth monitoring strategy was used throughout the process, and all models were trained from scratch and shared the same parameter value and Dice loss optimization. It was noted from Table 1 that the RDA-UNET model achieved 96.25% DSC, 96.34% precision, and 96.88% recall for the left kidney and 94.22% DSC, 95.34% precision, and 94.61% recall for the right kidney, which were better than other algorithms. The comparison between U-Net revealed that the use of BN greatly improved the segmentation performance.

The segmentation results of different models are shown in Figure 6. It was noted that compared with other algorithms, the RDA-UNET can segment the image more accurately and can effectively cope with changes in the shape of the kidney cysts.

### 3.2. Visualization of Results

#### 3.2.1. The User Interface

Figure 7 shows the user operation interface.  Figure 7(a) is the initial interface, which was mainly composed of three parts of the button for selecting the image, the button for segmenting, and the image display container. Clicking the button to select the image can load the image from the catalog to the interface.  Figure 7(b) is the screen displayed on the interface after the original CT image was loaded. To click the segmentation button, the system would automatically start the image segmentation, and the segmentation results were then displayed and saved.  Figure 7(c) shows the final segmentation results. When the segmentation was completed, the resulting image would be displayed. The red solid line is the contour of the kidney cyst depicted.

#### 3.2.2. Three-Dimensional Reconstruction Results

As shown in Figure 8, the CT image of a patient was segmented first, and then the segmentation results were fused. ITK-SNAP software was used to construct a three-dimensional image.

## 4. Discussion

The constantly accelerated life rhythm resulting from the development of the economy results in constantly increasing pressure, so more and more diseases occur, threatening the health of people. The kidney disease is a representative one and attracts more and more attention. With the widespread application of artificial intelligence technology in medical imaging, image segmentation technology based on deep learning has become a focus. Intelligent algorithm can effectively segment images to obtain detailed image data, providing reference for the clinical diagnosis and treatment. In this study, a deep-learning-based segmentation model, RDA-UNET, was designed based on the residual dual-attention module, and its performance was compared with FCN-8S, FCN-16S, U-Net, FCN-VGG10, and U-Net (+BN). The results showed that the loss function value of the RDA-UNET model attenuated and tended to converge in a short time, in line with the research results of Zheng et al. [19], who combined deep learning with marginal space learning (MSL) to construct a renal segmentation algorithm and found that the segmentation accuracy of the RDA-UNET model was higher than that of other traditional algorithms.

Finally, RDA-UNET was compared with FCN-8S, FCN-16S, U-Net, FCN-VGG10, and U-Net (+BN) models, factoring into different evaluation indicators. The results showed that the RDA-UNET model achieved 96.25% DSC, 96.34% precision, and 96.88% recall for the left kidney and 94.22% DSC, 95.34% precision, and 94.61% recall for the right kidney, which were better than other algorithms. Thong et al. introduced two transformation methods and proposed a simple depth segmentation model, which can enhance the segmentation of renal CT images [20]. Xia et al. designed a semantic segmentation model based on the SCNN and ResNet combined with SIFT flow transform, which achieved a good segmentation effect with a small proportion of detailed information [21]. Sharma et al. proposed a neural network model for the segmentation of multiple renal cysts based on the structure of the VGG network. However, the morphology of renal cysts would change greatly with renal disease, so the edge contour of renal cysts could not be well located [22]. The results confirmed that the RDA-UNET model constructed in this study had good application feasibility in intelligent segmentation of renal organs and quantitative evaluation of nephropathy.

## 5. Conclusion

In this study, RDA-UNET, a new segmentation model based on deep learning, was proposed to segment CT images of renal cysts. Through comparison with other kidney segmentation models in terms of Dice, precision, and recall, it proved that this model had obvious advantages in the segmentation of CT slice images of renal cysts. However, some limitations in the study should be noted. The sample size is small, which will reduce the power of the study. In the follow-up, an expanded sample size is necessary to strengthen the findings of the study. In conclusion, the RDA-UNET model has high accuracy in the segmentation of CT images of renal cysts, and the study provides a reference for the diagnosis and treatment of kidney diseases.

## Figures and Tables

**Figure 1:** RDA-UNET network structure.

**Figure 2:** RDA module structure.

**Figure 3:** Evaluation method.

**Figure 4:** The decay curve of the loss function.

**Figure 5:** Segmentation effect and the visualization (the first line is the segmentation result, the red line is manual labeling, and the blue line is the network segmentation result. The second line is the spatial attention mask generated by the last RDA module).

**Figure 6:** Segmentation results of different models. (a) Original image. (b) Manually annotated result. (c) RDA-UNET. (d) FCN-VGG10. (e) U-Net.

**Figure 7:** Schematic diagram of the user operation interface. (a) Initial interface. (b) Image loaded. (c) The result displayed.

**Figure 8:** Three-dimensional reconstruction of a CT image of renal cysts.

**Table 1:** Average value of the evaluation index of different deep network models on the test set (%).

Model		FCN-8S^[24]^	FCN-16S^[24]^	FCN-VGG10^[19]^	U-Net^[27]^	U-Net (+BN)	UNet++^[32]^	RDA-UNET
Left kidney	DSC	88.12	87.53	95.23	92.65	95.09	94.88	96.25
	Precision	89.25	87.22	96.45	92.48	95.67	95.22	96.34
	Recall	89.88	87.43	95.55	93.66	96.45	95.88	96.88

Right kidney	DSC	85.34	84.13	92.23	90.44	93.79	93.32	94.22
	Precision	87.83	84.23	95.88	91.67	94.67	95.11	95.34
	Recall	87.03	88.46	91.19	92.57	94.65	94.45	94.61

## Data Availability

The data used to support the findings of this study are available from the corresponding author upon request.
